This article has been retracted.

# Occupational Therapy and Prevention of Common Sports Injuries for Special Physical Training

**DOI:** 10.1155/2022/6227377

**Published:** 2022-07-05

**Authors:** Tao Lei, Yi Huang, Zhijuan Zhou

**Affiliations:** ^1^College of Physical Education Science, Hengyang Normal University, Hengyang Hunan 421001, China; ^2^School of Sports and Art, Hunan University of Medicine, Huaihua Hunan 418000, China

## Abstract

This paper provides an in-depth study of occupational therapy and the prevention of common sports injuries in special physical training. The issue of sports injuries and rehabilitation has always been a hot topic in special training. With the continuous development of sports, the increasing intensity of competition, and more stringent requirements for special techniques, the increase in difficulty and intensity of training has led to the increasing frequency of sports injuries, so how to prevent injuries in special physical training and rehabilitation and recovery of athletes after the injury is particularly important. Since the most common musculoskeletal injuries occur in the lower quadrant, this paper proposes a lower extremity functional test (LEFT) model as a means of identifying injury risk and guiding the implementation of training programs to prevent sports injuries. In this paper, a knee injury is used as an example, and an occupational therapy program of TCM physical therapy + aquatic rehabilitation is adopted for the already occurred sports injuries. Through interviews and clinical examinations of athletes, coaches, and medical personnel, this paper summarizes the sites, types, characteristics, and probability of occurrence of common sports injuries in special physical training. Experiments were conducted through clinical rehabilitation of common sports injuries with the addition of TCM manual massage. A series of effects of this modality on the rehabilitation of sports injuries were examined by monitoring physiological and biochemical indexes and by comparative analysis before and after testing physical function indexes using the Omega Wave system. Sports injuries are diverse. Traditional Chinese medicine physical therapy + water rehabilitation therapy is an effective physical therapy method. According to the relevant theories of traditional Chinese medicine treatment, diagnosis and treatment through meridians and related acupuncture points have significant curative effects. Traditional Chinese medicine, massage, and acupuncture have irreplaceable roles in the rehabilitation and treatment of sports injuries and can effectively improve and cure sports injuries.

## 1. Introduction

The problem of sports injuries is especially prominent among athletes of the same type with similar tactical levels and little difference in physical fitness [1]. The key to athletes' excellent performance lies in avoiding sports injuries as much as possible, detecting them in a timelier manner, and rehabilitating them faster and better. At the same time, this is also a problem that athletes themselves, coaches, and medical personnel must pay attention to and urgently need to solve in training and competition. In addition, sports injuries will also have a greater impact on the psychology of athletes, athletic status, and level of maintenance, becoming an obstacle on the road to high-level athletes [2]. The objective existence of sports injuries requires athletes to comply with the regularity and science of training content; otherwise, it is easy to lead to the occurrence of injuries and even affect the physical and mental health of athletes. Since sports injuries will inevitably occur in the daily training and competition of athletes, it is necessary to understand the causes of sports injuries and countermeasures, on the one hand, after the occurrence of injuries can be dealt with promptly and effective rehabilitation, on the other hand, to reduce or avoid sports injuries as much as possible, to minimize the adverse effects of sports injuries on the training and athletic level of athletes.

To break the existing pattern of achievement in the field of competitive sports, we should analyze the causes of the problems of nonadvantageous projects and compensate for the shortcomings while maintaining the traditional advantageous field projects, to promote the overall balanced development of each project and finally achieve a new situation of all-round development of each project. From the point of view of sports, our development and performance in physically demanding and fierce confrontation projects have been unsatisfactory, such as track and field and the three major ball games [3]. Therefore, we should follow the overall trend and future direction of international competitive sports development, study the successful experience of international first-class athletes in training and correctly grasp the laws of project training and development according to the actual situation, scientifically develop physical training, and then promote the overall development of other competitive elements such as skills, and combat energy.

The development of research and practice in the field of physical therapy rehabilitation in the United States gave rise to functional training, and subsequently, its training and methodological tools were introduced into the field of competitive sports [4]. In its subsequent development, functional training has received extensive attention from sports experts and scholars and front-line coaches, a lot of research has been conducted on its theoretical and practical aspects, and it has also been promoted vigorously.

Sports injury is a common injury problem in sports. Athletes need a lot of sports training and competition experience to improve their athletic ability and level, therefore, competitive sports and sports injuries have always gone hand in hand. Sports injuries have a great impact on the normal training of athletes, preventing athletes from creating good results in the competition, and even causing serious consequences for athletes to end their sports careers early [5]. Only by mastering the causes of sports injuries and formulating detailed prevention programs can the incidence of sports injuries be reduced; when sports injuries inevitably occur, good occupational therapy and rehabilitation training can help athletes recover their health as soon as possible [6]. The biggest enemy of an athlete is not a powerful opponent, but injury. Injuries and diseases not only restrict whether athletes can achieve better results but also affect the future direction of the sport. Therefore, it is of great practical significance to reduce the risk of athletes' injuries during special physical training and to improve the effect of sports injury rehabilitation treatment. This paper systematically studies the rehabilitation effect of traditional Chinese medicine physiotherapy + water rehabilitation on common injuries. On the one hand, it enables athletes and coaches to have a deeper understanding of the rehabilitation effect of traditional Chinese medicine physiotherapy + water rehabilitation on sports injuries, and on the other hand, it can provide a reference for athletes to formulate rehabilitation training plans after sports injuries.

## 2. Related Works

The meaning of sports injuries is that people in the process of sports, the occurrence of sports-related injuries and injuries. This kind of injury and injury is related to the sports project and has certain technical characteristics [7]. The injury and injury caused by sports often have a direct or indirect relationship with the characteristics of the sport itself (technology and tactical movements), the behavior of the sports subject (training level), objective conditions (sports environment, equipment, and equipment), and other factors. With the development of sports medicine, a comprehensive grasp and understanding of the possible physical injuries that may occur during sports are of great significance to the prevention of sports injuries [8]. As an important part of sports medicine, clinical work, and sports medicine discipline, a sports injury is of great value to enrich sports medicine theory and practice. The causes of athletes' sports injuries include poor physical condition, substandard technical movements, insufficient self-protection ability, inadequate preparation activities before sports, and improper training and participation organization. Lin et al. mentioned in the hot spots and analysis of innovative research on sports injuries in the United States that one of the causes of sports injuries is overuse injuries, overuse injuries are injuries caused by long-term repetitive movements that cause pathological reactions in a certain part of the body, and such injuries are most frequently studied in long-distance runners [9]. One survey estimated that the probability of injury due to long-term repetitive loading was as high as 79% in middle and long-distance runners and 90% in marathon runners. Sports injuries do not arise from a single cause, it contains the technical characteristics of the sport, the field environment, clothing, and the individual physiological and psychological conditions of the athlete now.

Sports injury prevention is like the tertiary prevention of disease proposed by the World Health Organization (WHO), in which primary prevention, i.e., etiological prevention, is the intervention to target the cause of injury before it occurs, which is the fundamental measure to prevent sports injury and eliminate the cause of injury and is also the most active and effective preventive measure among the tertiary prevention. For primary prevention of sports injuries, Hung and Fong proposed a model that describes the incidence and severity of injuries and emphasizes the identification of injury risk factors and causal mechanisms through prospective studies [10]. Bezhentseva also suggested that it is not enough to determine the correlation between motor screening test results and sports injuries through prospective studies, but also to suggest how to change the risk factors associated with motor screening test results based on them and verify whether they are effective in reducing the risk of sports injuries [11].

Physical therapy is a term that originated from ancient Greek and originally meant “to heal by the power of nature.” It uses various physical factors to prevent disease. Physical factors include both natural and manufactured behaviors [12]. Natural physical factors refer to the various physical factors in nature that have medical and health care functions, such as air, seawater, sunlight, and mineral springs. Artificial physical factors refer to various physical energies obtained through artificial methods, such as light, electricity, magnetism, sound, and heat. With the continuous development of modern science and technology, the content and scope of physical therapy can be expanded according to the condition of various parts of the patient's body (such as joint mobility and muscle atrophy). In a study of the characteristics and psychological impact of sports injuries in outstanding athletes of different sports, Bartnovskay et al. found that the nature and causes of sports injuries in professional athletes were related to the sports they were engaged in [13]. This article adopts traditional Chinese medicine physical therapy + water rehabilitation therapy as an occupational treatment plan for sports injuries. First, it can reduce the side effects caused by the intake of drugs by athletes with sports injuries and can shorten the recovery period of athletes. At the same time, the occupational therapy program has positive significance for athletes, coaches, and the normal progress of various competitions.

## 3. Method

### 3.1. Study Design

The most common musculoskeletal sports injuries occur in the lower quadrant (LQ), and for the prevention of common sports injuries in special physical training, the lower extremity functional test (LEFT) is proposed in this paper, with the following ideas.

- Determine the action tasks and scoring criteria for LEFT
- Reliability tests were conducted on the LEFT, including interrater reliability, intrarater reliability, and subject retest reliability
- Based on b, predictive validity tests were performed for LEFT. A retrospective cohort study was conducted to determine whether the LEFT could discriminate between subjects with and without a history of LQ injury; a prospective cohort study was conducted to determine whether the LEFT could effectively predict the risk of LQ sports injury and to establish a regression equation that could calculate the risk of injury; finally, a cross-sectional study was used to investigate the relationship between LEFT test results and LQ injury risk factors, such as balance, muscle strength, and flexibility [14]. Finally, a cross-sectional study was conducted to investigate the relationship between LEFT test results and LQ injury risk factors such as balance, strength, and flexibility, and to establish the basis for developing targeted training

For the sports injuries that have occurred, this paper proposes an occupational therapy model with TCM physical therapy + aquatic rehabilitation.

### 3.2. Participants

Athletes with a history of knee injury who participated in municipal youth soccer training were used in this study. For this study, youth soccer players (aged 14-19 years) from municipal sports schools and high-level clubs were screened for lower limb injuries, and athletes who had lower limb sports injuries and were seen at the National Sports General Administration Sports Hospital were evaluated for lower limb function and administered appropriate rehabilitation strategies. The athletes were randomly divided into an experimental group and an injury control group, with 12 athletes in each group. The experimental group was given targeted rehabilitation treatment and lower extremity functional training, while the rest of the daily training and life was the same as the control group, and the injury control group maintained the same daily training and life.

Entry requirements are (1) soccer-specific level 2 or above athletes, (2) knee injury and the injury time has been more than 6 months, and (3) currently no serious discomfort, can normally participate in classes, training, games, and other activities.

Exclusion criteria were (1) athletes in the acute injury and rehabilitation phases, (2) athletes who were otherwise unable to participate in normal classes, training, games, and other activities, and (3) athletes who did not wish to participate in the study. Another 12 soccer players without lower extremity sports injuries matched for age, gender, training years, and athlete level were selected as healthy controls to compare the impaired knee muscle strength and function of the injured athletes and the degree of recovery after training.

### 3.3. Measures

1. *Data Extraction and Quality Analysis*. Data collection was conducted through a predesigned data extraction form, with two researchers working in groups to extract data separately and cross-check all data included in the studies. Information extracted from each study included: general information about the literature (e.g., first author and year of publication); trial design, study population (e.g., occupations such as sports, military/fire, age, and sample size); injury definition, and method of judgment; injury calculation (e.g., incidence rate proportion, incidence, and prevalence); risk factors; and outcomes (e.g., significance and nonsignificance) including reliability indicators, risk indicators (e.g. mean difference, correlation, OR, incidence rate ratio (IRR), and risk ratio (RR)), and diagnostic accuracy (e.g., area under the subject characteristic curve AUC, sensitivity, specificity, negative predictive value, positive predictive value, positive or negative likelihood ratio).

The quality of evidence was assessed based on criteria of internal validity (study design, quality reporting, selection and misclassification bias, and potential confounding) and external validity (generalizability). The downs and black (DB) quality assessment tool was used to scoring each study based on each criterion, with a total score of 32 points per study (10 points for reporting, 3 points for external validity, 7 points for bias, 6 points for confounding, and 5 points for weighting) [15]. The level of evidence for each study was classified according to the Oxford Centre for Evidence-Based Medicine (OCEBM) 2009 model, and levels 1a, 2a, 3a (systematic reviews), 4 (case series), and 5 (opinion-based papers) were excluded according to the study's exclusion criteria. Differences in DB scores or OCEBM classifications were first agreed upon by the two researchers who scored the study, and in case of disputes, the subject leader will decide. The key to achieving excellent results in mobilization is to avoid sports injuries as much as possible, to detect sports injuries in a timely manner, and to recover faster and better.

(2) In verifying the reliability of the lower limb functional evaluation scale, the Cronbach's alpha coefficient of the functional evaluation scale was verified using SPSS 19.0; statistical aspects of the data on the epidemic disease survey of youth soccer players were statistically analyzed using Microsoft Excel 2010 to provide a basis for article writing, to maximize the value of the data and uncover. We aim to maximize the value of the data and explore the value behind the data

### 3.4. Design

#### 3.4.1. Manipulative Massage for Rehabilitation of Joint Injuries

Joint injuries in special physical training are mostly knee injuries and ankle injuries. In this study, knee injuries were mostly injuries to the femoral ankle, tibial plateau, patella, and its surrounding synovial membrane, joint capsule, and articular cartilage [16]. Ankle injuries were mostly sprains and ligament strains caused by internal and external rotation or inversion of the foot and injuries to the articular cartilage. The role of manual massage is to improve the blood supply to the joint parts and soothe the meridians to relieve and prevent tendon adhesions, which is conducive to the recovery of the athletes' joint mobility and extension and flexion so that the normal activities and functions of the athletes' joints can be guaranteed.

Massage techniques.

1. *Rubbing*. Use the palm of the large fissure to press the injury site for 1 ~ 2 minutes, acute injury should be cold or hot compress treatment before massage rehabilitation, and massage techniques are not recommended for immediate rehabilitation
2. *Buckling*. Use your thumb to buckle inward on the painful spot for 3 to 4 minutes, to the degree of pain or soreness
3. *Plucking*. For knee injuries only, pluck 10 times from side to side with the thumb on the muscle attachment points around the injury site
4. *Rotational Pulling*. For ankle injuries only, one hand immobilizes the ankle and presses the painful point with the thumb while the other hand pulls the ankle outward and rotates it accordingly
5. *Point*. Press with the thumb for 30 seconds to 1 minute at the Foot San Li, Blood Sea, Knee Yang Guan, Yang Ling Quan, Wei Zhong, Wei Yang, Cheng Shan, Cheng Tendon, and Kun Lun points, respectively

#### 3.4.2. Water Rehabilitation Means for Knee Injuries

Developing multidirectional movement of all muscle groups around the knee is the key to recovery. The injured area can be rehabilitated through water exercise because of the water's stress-reducing effect on the knee joint, which makes water the perfect vehicle for recovery activities from knee trauma or knee surgery [17]. In addition, any knee injury can be extremely painful and potentially disabling, so effective pain management is also important to the overall rehabilitation process. It can effectively relieve the heart fatigue and central nervous fatigue caused by the disorder of the vagus nerve regulation system and the sympathetic nerve regulation system and greatly relieve the physical fatigue and the reduction of the recovery ability of athletes.

By interviewing 10 experts, the experts were asked to evaluate the effectiveness of water rehabilitation tools for knee injuries by using the assignment method with a score of 10 out of 10, and the average value was taken as the evaluation score of each rehabilitation tool, with lower scores indicating lower effectiveness.

#### 3.4.3. LEFT Action Design

In this paper, we designed a movement screen designed to predict the risk of LQ injury. The test consists of 5 movement tasks involving different movement patterns, planes, orientations, and intensities, encompassing both structural and functional tests, with movement quality (MQ) and symptom score (SS) results. These tasks were (A) Single-leg stand, trunk extension, neck rotation (L 1); (B) Single-leg stance with trunk rotation and hip flexion (L 2); (C) Single-leg squat with knee extension and heel lift (L 3); (D) Four-way jump (L 4); (E) Single-leg jump with half turn (L 5).

The MQ of LEFT has a total score of 100 points, 50 points for the left, and 50 points for the right side, with higher scores representing better movement quality. The quality score of each movement is composed of the number of completions, continuity, and technical points, accounting for 3, 2, and 5 points, respectively, with a total of 10 points.

(1) $$\begin{array}{c} Vas\geq N,0\leq N\leq 10. \end{array}$$

The total SS score of LEFT is 100, with 50 points on the left and 50 points on the right. Higher scores represent less (mild) symptoms such as pain, numbness, and pinching during the movements, and a full score means that these movements do not cause any symptoms, while a score of 0 represents severe pain (*Vas* ≥ 7) or another severe discomfort that prevents completion of the movements. The score is composed of the raw score and the adjustment factor. If pain, weakness, numbness, and pinching occur simultaneously, the lowest symptom score minus the adjustment factor is taken; otherwise, only the raw score is recorded.

The concepts of reliability and validity were first derived from psychological research on the reliability and validity of tests. Reliability refers to the stability and consistency of the measurement results, i.e., whether the results obtained by the measurement instrument are stable. Commonly used reliability indicators include interrater reliability, intrarater reliability, and retest reliability. Validity refers to validity or accuracy, i.e., the degree to which a measurement instrument can measure the trait it is intended to measure [18]. The higher the validity, the better the results show the true characteristics of the object to be measured. Common validity indicators include calibration validity, discriminant validity, predictive validity, and content validity.

In this study, we determined the theoretical framework for the development of LEFT based on the results of previous movement screening studies, identified 5 movements of LEFT using domestic and international expert discussions, and developed the movement quality and symptom scoring criteria of LEFT. To further clarify the reliability and validity of the LEFT, identify risk factors through the LEFT test results, and establish a basis for developing targeted training programs, we conducted the following four tests to comprehensively evaluate the reliability (interrater reliability, intrarater reliability, and subject retest reliability) and predictive validity of the LEFT.

### 3.5. Analysis

A total of 200 questionnaires were distributed in this trial and 126 were returned, with 88 completed and valid questionnaires. According to the inclusion and exclusion conditions, 30 people with chronic knee or ankle injuries were screened as subjects. Thirteen people in the experimental group had mild injuries, and two people had moderate injuries. The average duration of injury was 0.9 years, and the average duration of exercise was 7.5 years. In the control group, 10 people also had a mild injury (no swelling of the muscles around the knee joint, slight pain in the lower part of the inner and outer ankle or the tibiofibular ligament, no abnormal walking, and slight discomfort after strenuous running and jumping), 5 people had a moderate injury (discomfort after strenuous knee activities, slight weakness during exercise, or increased pain by passively pulling the ankle joint or pulling the injured collateral ligament), the average injury time was 1 year, and the average exercise time was 8.5 years. From the analysis of the above data, there was no significant difference between the experimental group and the control group subjects in terms of basic data such as playing position, age, height, and weight *p* > 0.05.

The occurrence of sports injuries is not a single cause, but includes the technical characteristics of sports, venue environment, clothing, and the current physical and psychological conditions of athletes. The occurrence of sports injuries is often not accidental, there must be internal and external causes, a fuller understanding of the causes of sports injuries can be better to carry out rehabilitation treatment, for sports injury rehabilitation treatment to find the premise of targeted direction. Comprehensive domestic reasons for the occurrence of sports injuries are combined with the investigation of the causes of injury to city soccer players, and the causes of sports injuries can be broadly summarized as poor training levels, training method errors, fatigue, and climate factors, which are four aspects, see Table 1.

## 4. Results

### 4.1. Analysis of the Rehabilitation Effect of Manual Massage on Joint Injury

In the analysis and comparison of the results of physical function index testing of municipal soccer players using the Omega Wave instrument, it can be seen that manipulative rehabilitation has a good recovery effect on the vagal regulatory system and sympathetic regulatory system of the athletes, can effectively relieve the cardiac fatigue and central nervous fatigue caused by the dysregulation of the vagal regulatory system and sympathetic regulatory system, which greatly relieves the athletes' physical fatigue and reduced recovery ability, and has a significant improvement effect on the heart's inability to withstand heavy exercise caused by nervous tension and nonperiodic factors; at the same time, it can restore the athletes' cardiopulmonary regulation system. On the one hand, it can be treated in time and effectively recovered after the injury occurs, on the other hand, reduce or avoid sports injuries as much as possible, and minimize the adverse effects of sports injuries on the training and competition level of athletes.

In the analysis of the monitoring results of the physiological and biochemical indexes of the city soccer players, it can be seen that the manipulative rehabilitation has a significant alleviating effect on the elevation of serum creatine enzyme and blood urea nitrogen, and the decrease of hemoglobin and serum testosterone in the body of the athletes caused by a sports injury or high intensity and high load sports training effectively avoids the low immunity caused by a sports injury or sports fatigue [19]. Through the rehabilitation treatment of manual massage, the stability and recovery of various physiological and biochemical indexes in the athletes' organism have been significantly improved. While the athletes' physical function is stable and the recovery effect is good, the low adaptability to sports load and physical discomfort caused by sports injury of the athletes are effectively improved. It significantly improves the effect of sports injury rehabilitation treatment and enables athletes to recover faster and better to the preinjury state and level after the occurrence of sports injury.

### 4.2. Results of Water Rehabilitation Tools for Knee Injuries

Ligament injuries to the knee are one of the most common knee injuries that occur in athletes of all ages and professions. This injury usually results from a direct bending of the outside of the knee in sports such as soccer or rugby [20]. For example, a sudden turn inside the knee can cause this injury in activities like skiing or soccer with undercutting movements. Due to the gravity-free environment of the water, aquatic therapy is the perfect modality to recover from ligament injuries. There is no weight placed on the joint in the water, and the weight of the leg is effectively supported by the buoyancy of the water. Initially, knee flexion (bending due to gravity) can be avoided. The focus of an underwater rehabilitation program should be to consolidate the strengthening of all muscle groups around the knee, ankle, and hip.

The main goal of knee treatment and rehabilitation is to allow the injured structure to heal without losing the mechanical stability of the knee joint. The results of the evaluation of the effectiveness of rehabilitation tools in water for knee injuries are shown in Figure 1.

As can be seen from the chart above, the effectiveness scores of water rehabilitation methods for knee injuries are all above 8, and the most effective rehabilitation methods are knee lift and lunge walking exercises. The goals and principles of rehabilitation for meniscal, ligament, articular cartilage, and cruciate ligament injuries are similar. The exercises used during the rehabilitation period are essentially the same for all types of knee injuries.

### 4.3. Reliability and Validity Test Results of LEFT

Twenty subjects (age 22.0 ± 1.0 years; height 176.1 ± 3.5 cm; weight 69.3 ± 4.9 kg) completed this test. Subject demographic information is shown in Table 2. 3 raters were second-year master's students in exercise science-related disciplines.

The results of the ANOVA showed that there was no statistical difference between the scores of the different raters participating in the LEFT composite MQ reliability study; there was also no statistical difference between the two video scores of the same raters (*F* = 0.353; *p* = 0.705; *F* = 0.708, *p* = 0.404); there was no statistical difference between the two LEFT test MQ scores of the subjects (*F* = 0.156; *p* = 0.679), as shown in Figure 2. Interrater reliability, intrarater reliability, and subject retest reliability were excellent.

Binary logistic regression analysis showed that the LEFT test results MQ (OR = 0.916, *p* = 0.004) and SS (OR = 0.919, *p* = 0.003) were both associated with LQ impairment, with subjects with 1-unit higher MQ being 0.916 times more likely to have LQ impairment than subjects with 1-unit lower MQ, and subjects with 1-unit higher SS being 0.919 times more likely to have LQ impairment than subjects with 1-unit lower SS, *R*2 = 0.312 (adjusted *R*2 = 0.453). 0.919 times more likely than subjects with SS one unit lower, *R*2 = 0.312 (adjusted *R*2 = 0.453). Thus, MQ and SS can be used as independent predictors of the risk of LQ injury, as shown in Figure 3.

When MQ and SS were used as independent predictors to predict the risk of LQ injury, the area under the ROC curve was AUC = 0.772 (*p* = 0.001, 95% CI: 0.653-0.891) and AUC = 0.771 (*p* = 0.001, 95% CI: 0.638-0.905), respectively. When MQ and SS were used together as predictors, AUC = 0.853 (*p* = 0.001, 95% CI: 0.754-0.953), indicating that 85.3% of LQ injuries could be correctly predicted by LEFT. The ROC curves of MQ and SS to differentiate LQ injury history are shown in Figure 4.

The relationship between LEFT test results and LQ injury was analyzed by a prospective cohort design, regression equations were established, and the accuracy of prediction was determined by ROC curves. The results showed that MQ and SS could be used as independent predictors of LQ injury, respectively, and the combination of MQ and SS as predictors could improve the accuracy of prediction. LEFT showed good predictive validity when predicting the risk of LQ injury and can be a valid test tool for calculating the risk of LQ injury based on the regression equation.

## 5. Discussion

Sports injuries occur mostly in training and competition; sports injuries occur mostly in the winter season; athletes have less severe injuries, mostly mild, and moderate injuries, but there are more chronic injuries, the number of disease duration of more than a year accounted for most, while the injury is mostly nonopen closed injury. Many athletes' injuries cannot be recovered overnight, as the saying goes, “sickness comes like a mountain, dispel the disease like a silk.” For many chronic sports injuries and overuse injuries, TCM physical therapy is highly favored because of its unique theory of Chinese Tuina and the valuable experience of traditional Chinese medicine. TCM physiotherapy is very effective in treating many chronic injuries and overuse injuries in special physical training through manipulation of tendons and points. Sports injuries are diverse, and rehabilitation therapy in TCM is effective as an effective physical treatment method through meridians and related acupuncture points according to the relevant theories of TCM treatment. Chinese medicine, tui na, and acupuncture have an irreplaceable role in the rehabilitation process of sports injuries and can effectively improve and cure sports injuries.

## 6. Conclusion

The LEFT model is proposed in this paper, and the reliability and validity tests show that LEFT is a stable, reliable, and valid measurement tool that can effectively identify people with a history of lower quadrant injury, and more importantly, it can accurately predict the risk of lower quadrant injury through the established regression equation, which is one of the very best tools for sports injury prevention. The effectiveness of TCM physiotherapy + aquatic rehabilitation for knee rehabilitation is proposed and validated for sports injuries that have already occurred. TCM physical therapy + aquatic rehabilitation significantly improved extension range, flexion range, pain scores, knee flexor muscle strength, knee scores, and walking ability in patients with knee injuries. However, there was no significant improvement in improving the ability to perform activities of daily living, and more high-quality samples are still needed for further studies. In the future work, we can start from this aspect to conduct more in-depth and meticulous research, so that physical therapy can penetrate into all aspects of physical training and give eternal care throughout the whole process.

## Figures and Tables

**Figure 1:** Results of the evaluation of the effectiveness of in-water rehabilitation tools for knee injuries.

**Figure 2:** Composite MQ interrater reliability and intrarater reliability.

**Figure 3:** Binary logistic regression analysis of MQ and SS as predictor variables.

**Figure 4:** ROC curves of MQ and SS to distinguish the damage history of LQ.

**Table 1:** Causes of athletic injuries in athletes.

Causes of sports injuries	Number of people	Percentage
Poor training	6	20.00%
Wrong training method	8	26.67%
Physical fatigue	12	40.00%
Climate factor	4	13.33%
Total	30	100.00%

**Table 2:** Trial 1 subject demographic information.

Subject/(unit)	Mean	Standard deviation	Scope
Age/(years)	22.0	±1.0	21-23
Height/(cm)	176.1	±3.5	172-180
Weight/(kg)	69.3	±4.9	64-75
Exercise frequency/(times/week)	5.3	±0.2	5-6

## Data Availability

The data used to support the findings of this study are available from the corresponding author upon request.
